The article "Endoplasmic Reticulum Stress in Bone Metastases" was published in 2020. Journal: Front Oncol.

# Endoplasmic Reticulum Stress in Bone Metastases

**DOI:** 10.3389/fonc.2020.01100

**Published:** 2020-07-24

**Authors:** Longyong Xu, Weijie Zhang, Xiang H.-F. Zhang, Xi Chen

**Affiliations:** ^1^Department of Molecular and Cellular Biology, Baylor College of Medicine, Houston, TX, United States; ^2^Lester and Sue Smith Breast Center, Baylor College of Medicine, Houston, TX, United States; ^3^Dan L. Duncan Cancer Center, Baylor College of Medicine, Houston, TX, United States

**Keywords:** bone metastases, seed and soil, metastatic niche, ER stress, unfolded protein response, immunotherapy

## Abstract

Metastases—the spreading of cancer cells from primary tumors to distant organs, including bone—is often incurable and is the major cause of morbidity in cancer patients. Understanding how cancer cells acquire the ability to colonize to bone and become overt metastases is critical to identify new therapeutic targets and develop new therapies against bone metastases. Recent reports indicate that the endoplasmic reticulum (ER) stress and, as its consequence, the unfolded protein response (UPR) is activated during metastatic dissemination. However, their roles in this process remain largely unknown. In this review, we discuss the recent progress on evaluating the tumorigenic, immunoregulatory and metastatic effects of ER stress and the UPR on bone metastases. We explore new opportunities to translate this knowledge into potential therapeutic strategies for patients with bone metastases.

## Introduction

Bone is a frequent site of cancer metastases, and skeletal metastasis is much more common than the primary bone cancers (1). Metastatic spread of primary tumor cells to bone tissues comprises the following multiple-step cascade: (1) local invasion at the primary site; (2) intravasation; (3) survival in circulation; (4) arrest at distant organ sites; (5) extravasation to enter the parenchymal tissues of distant organs; (6) survival in the new microenvironment; and (7) proliferation to form macroscopic, clinically detectable secondary tumors, which is the step that eventually leads to morbidity (Figure 1) (2–4). Considerable research efforts have demonstrated that both intrinsic traits of cancer cells (the seeds) and the unique bone microenvironmental factors (the soil) contribute to the development of bone metastases (1, 3, 5–7). These efforts have led to approved treatment on bone metastases, exemplified by the introduction of bisphosphonates and denosumab (8–10). Meanwhile, several clinical trials are on-going based on the knowledge from these efforts. Further studies aim to understanding the molecular basis for each step of bone metastasis will be instrumental to manage the bone metastasis.

**Figure 1:** The multistep process from primary tumor to bone metastasis. During metastatic progression, tumor cells leave their primary site via local invasion into the surrounding tumor-associated stroma, followed by tumor cell intravasation into the blood and lymph vasculature. Once in the vasculature, tumor cells interact with neutrophils and NK cells, which regulate their survival in the circulation. These steps above are mostly common in metastasis to different distant organs. The extravasation of cancer cells from the blood vasculature into the bone marrow can occur very early. After extravasation, colonizing cancer cells must develop survival mechanisms to adapt to the local microenvironment and various treatment. This includes dormancy, interacting with (pre)metastatic niche cells (e.g., osteoblasts and osteoclasts), and resistance to immunity. Of those cells that survived, some will be reactivated after years, even decades, to form macrometastasis.

Tumor cells endure intrinsic (oncogenic) and extrinsic environmental stresses during metastatic dissemination (11). These stresses can either increase the protein synthesis, overwhelming the protein folding capacity of the endoplasmic reticulum (ER) or directly disrupt ER protein folding. This leads to the accumulation of unfolded and misfolded proteins (known as ER stress) (12, 13). An adaptive mechanism, termed the unfolded protein response (UPR), is consequently initiated by transmembrane sensors on the ER upon detection of ER stress to restore ER homeostasis (14). Multiple functions of the UPR in the development of primary tumors have been extensively studied, and targeting the UPR has been shown to be an effective therapeutic strategy in multiple cancers (15–28). However, its role in metastases remain far less documented. In this review, we will discuss the mechanisms of the UPR in tumor progression and its potential implications in bone metastases.

## Bone Metastases

The relative incidence, median survival, and effect on bone homeostasis (osteolytic, osteoblastic, or mixed) of bone metastases vary greatly among different cancer types (Table 1) (1, 29, 30). Bone metastases are associated with multiple skeletal complications, including bone pain, impaired mobility, pathologic fractures, nerve compression, bone marrow aplasia, and hypercalcemia (31). The clinical detection of metastases may be a late event of disease progression; although, the dissemination to bone may occur early. Disseminated tumor cells (DTCs) can be detected in the bone marrow of patients and in mouse models even without the invasive diseases (32–38). However, because many more DTCs than macrometastases are present in the bone marrow in both patients and mouse models, it remains unclear whether these early DTCs ultimately cause metastatic outgrowth or if they are simply bystanders during the metastatic process (5, 9). Nevertheless, it is clear that the presence of DTCs in bone marrow is associated with poor prognosis and predicts eventual metastases to the bone as well as other organs (39–43). The microenvironment in primary tumors contribute to the selection of secondary tumors in bone. For example, cancer-associated fibroblasts select Src-hyperactivated bone metastatic seeds in triple-negative breast cancers (TNBC) (44). Meanwhile, premetastatic niches in the bone microenvironment are actively formed by secreted factors and/or exosomes from the primary tumor prior to DTC seeding (5, 45, 46). Upon arrival at the bone, DTCs that survive the hostile environment interact with the bone resident cells, forming the metastatic niche that determines the fate of DTCs (dormant, reactivated, or drug resistant) (5, 7, 9, 47).

**Table 1:** Incidence of bone metastases in cancer (1).

**Primary cancer type**	**Relative incidence**	**Median survival (months)**	**Five-year survival rate**	**Impact to bone homeostasis**
Breast	65–75%	19–25	20%	Mixed
Prostate	65–75%	12–53	25%	Osteoblastic
Lung	30–40%	6	<5%	Osteolytic (NSCLC) Osteoblastic (SCLC)
Thyroid	40–60%	48	40%	Mixed
Bladder	40%	6–9	3%	NA
Renal	20–25%	6–12	10%	Osteolytic
Melanoma	14–45%	<6	<5%	Osteolytic

*NSCLC, non-small-cell lung cancer; SCLC, small-cell lung cancer*.

## ER Stress and the UPR

The ER is the major organelle in eukaryotic cells responsible for intracellular Ca^2+^ homeostasis, lipid biosynthesis, and the folding of membrane and secreted proteins (14, 48–52). Protein folding in the ER is precisely regulated and highly sensitive to alterations in the protein load, mutations that affect the folding process, and the ER folding environment (e.g., redox state, nutrient status, and Ca^2+^ levels) (49, 53). The accumulation of unfolded or misfolded proteins in the ER causes ER stress, which can be detected and resolved by the UPR (48, 51, 54–57). There are three major UPR signaling branches named after their transmembrane sensors: (1) inositol-requiring enzyme 1α (IRE1α, encoded by *ERN1*), (2) PKR-like ER kinase (PERK, encoded by *EIF2AK3*), and (3) activating transcription factor 6α (ATF6α, encoded by *ATF6*) (58) (Figure 2). All of these three sensors are activated upon the dissociation of the binding immunoglobin protein (BiP, encode by *HSPA5*) (59) or by the direct binding of unfolded proteins (60, 61) under ER stress.

**Figure 2:** Overview of the mammalian UPR. The three ER resident sensors (IRE1α, PERK, and ATF6) transduce information about the protein folding status of the ER to the cytosol and nucleus to restore the protein folding capacity. Under normal conditions, the sensors are inactivated by binding to the chaperone BiP. Under ER stress conditions, the sensors are activated by BiP dissociation and/or direct misfolded protein binding. Each pathway uses a different mechanism for signal transduction upon activation. IRE1α dimerizes, autophosphorylates, and triggers its RNase activity. This leads to the splicing of the XBP1 mRNA to produce an active transcription factor, spliced XBP1 (XBP1s). XBP1s induces the transcription of the genes encoding protein chaperones, ERAD, and phospholipid synthesis. The RNase activity of IRE1α also degrades certain mRNAs through RIDD. Activated IRE1α can activate the JNK, p38, ERK, and NF-kB pathways, thus playing an XBP1-independent role to modulate diverse cellular responses. Upon activation, PERK phosphorylates eIF2α, leading to global translational attenuation while selectively mediating translation of *ATF4*. In turn, ATF4 induces the expression of genes involved in amino acid metabolism, proapoptotic factor DDIT3/CHOP, and antioxidant responses (HO1). PERK also phosphorylates and stabilizes NRF2, a transcription factor involved in redox metabolism. ATF6 is transported to the Golgi apparatus under ER stress, where it is processed by S1P and S2P, releasing its cytosolic domain fragment as a transcription factor. ATF6 activates genes encoding protein chaperones, ERAD components, *and XBP1*. Abbreviations: ATF, activating transcription factor; BiP, binding immunoglobulin protein; *DDIT3*, DNA damage inducible transcript 3; eIF2α, eukaryotic translation initiation factor 2 subunit 1; ER, endoplasmic reticulum; ERAD, ER-associated protein degradation; HO1, heme oxygenase 1; IRE1α, inositol-requiring enzyme 1α; JNK, c-Jun N-terminal kinase; NF-kB, nuclear factor kappa light-chain enhancer of activated B cells; NRF2, NF-E2-related factor 2; PERK, PKR-like ER kinase; RIDD, regulated IRE1α dependent decay of mRNA; S1P and S2P, site 1 and site 2 proteases; UPR, unfolded protein response.

IRE1α is the most evolutionarily conserved branch of the UPR (62, 63). It is a bifunctional transmembrane kinase/endoribonuclease that dimerizes, and autophosphorylates upon luminal activation and then specifically cleaves 26 nucleotides from cytoplasmic X-box binding protein 1 (*XBP1*) mRNA (*Hac1* in yeast) (54, 55, 64–66). This is the first step of a cytoplasmic splicing event that creates an active form of the transcription factor XBP1s which, among its various functions activates multiple ER quality control genes to enhance the protein folding capacity of the ER to reduce the misfolded proteins there. Meanwhile, activated IRE1α also degrades certain ER-localized cytoplasmic mRNAs in a process known as regulated IRE1-dependent decay (RIDD) to reduce the number of proteins entering the ER (67, 68). By interacting with different adaptor and modulator proteins, IER1α can also activate the JNK, ERK, p38, and NF-kB pathways (69–71).

PERK is a serine/threonine kinase, and its best characterized substrate is eIF2α (72). PERK-dependent phosphorylation of eIF2α reduces the protein load into the ER by inhibiting the 5′ cap-dependent translation, while selectively increasing the translation of ATF4. ATF4 subsequently activates multiple genes involved in the regulation of autophagy, amino acid metabolism, and antioxidant responses (73–75).

Under ER stress, ATF6 is translocated to the Golgi apparatus, where it is cleaved by site 1 protease (S1P) and S2P, releasing the cytoplasmic transcription factor fragment (76). ATF6 activates genes that are involved in protein folding in the ER. Collectively, the consequences of UPR activation—pro-survival or pro-apoptotic—depend on the duration and intensity of the stress stimuli (14, 15, 20, 51, 53, 56).

## The UPR in Premetastatic Niche Formation

Survival and outgrowth of tumor cells in distant organs depend on their interaction with the microenvironment of the distal site (5–7). Several fundamental discoveries have revealed that cancer cells can remotely reprogram the microenvironments in distant organs to facilitate the later colonization, survival, and growth in a process termed prometastatic niche (PMN) formation (45, 46, 77). In the context of bone metastases, lysyl oxidase (LOX) is secreted by estrogen receptor–negative (ER^−^) breast tumors and mediates PMN formation in the bone (45). Hypoxia signature is correlated with increased risk of bone metastases, particularly in ER^−^ breast tumors. Cox et al. found LOX is highly expressed in bone-tropic MDA-MB-231 subline 1833-BoT cells and is associated with bone tropism in ER^−^ breast tumors. LOX secreted by the hypoxic primary tumor leads to the formation of premetastatic osteolytic lesions and promotes bone metastatic burden in a 4T1-BALB/c mouse model. The expression of *LOX* is induced by hypoxia inducible factor (HIF) under hypoxic conditions (45). Meanwhile, the UPR is known to be induced by hypoxia (15). Further study demonstrated that XBP1s interacts with HIF1α and is required for the upregulation of HIF1α-mediated hypoxia response pathway genes in TNBC tumors (18). This study implies that XBP1s may directly regulate the expression of *LOX* under hypoxic conditions. Indeed, XBP1 activates *LOX* expression in lung adenocarcinoma cells to promote the cell growth (78). Thus, the increased secretion of LOX in hypoxic tumors may be due to the activation of the UPR. It is compelling to note that blocking the IRE1a-XBP1 pathway may simultaneously inhibit the growth of both the primary TNBC tumors and bone metastases. Additional work will be required to test the universality of UPR involvement in the PMN formation during bone metastasis.

## Role of the UPR on the Survival of Circulating Tumor Cells

In the vasculature, circulating tumor cells (CTCs) encounter various stresses, including the loss of extracellular matrix (ECM) detachment, oxidative stress, innate immune response, and physical shear force (3, 79, 80). Normally, cells undergo apoptosis when they lose contact with their ECM or neighboring cells. This specific type of apoptosis, termed anoikis, prevents adherent-independent cell growth, attachment to an inappropriate matrix, and thus colonization of distant organs (79, 80). Multiple studies suggest that the PERK-eIF2α branch of the UPR inhibits anoikis and is required for tumors to invade and metastasize (81–83). The PERK-eIF2α pathway was shown to activate in suspension-cultured MCF10A cells and sustains MCF10A cell survival (81). Cells that undergo epithelial-to-mesenchymal transition (EMT) are highly secretory, and the PERK axis of the UPR was found to be selectively activated (82). In addition, the inhibition of PERK compromised the ability of EMT cells to form tumorspheres and migrate in transwell assays (82). Human melanoma cells experience higher levels of oxidative stress in the circulation and distant tissues than in primary tumors (84). To manage such oxidative stress, metastasizing melanomas undergo reversible metabolic adaptations, including the synthesis of antioxidants, to survive and eventually metastasize to distant sites. A previous study (83) showed that the PERK downstream transcription factor ATF4 and NRF2, which is stabilized by PERK (85), activate the expression of major antioxidant enzyme heme oxygenase 1 (HO-1), and therefore protect the detached cells from oxidative stress.

CTCs are also vulnerable to immune attacks by innate immune cells, notably NK cells (86, 87). In contrast to NK cells, neutrophils seem to protect CTCs and favor the metastatic spreading (4, 88). The functions of the IRE1α-XBP1 branch during the CTC stage are complicated (89–92). On the one hand, XBP1s promotes NK cell proliferation and positively regulates cytolytic activity of NK cells (89, 91, 92). On the other hand, XBP1 stimulates the expression of lectin-type oxidized LDL receptor 1 (LOX-1) in human neutrophils and transforms them into immunosuppressive cells, possibly promoting CTC survival (90). Overall, the PERK pathway could promote CTC survival by inhibiting anoikis and oxidative stress. Further *in vivo* studies are necessary to evaluate the overall effect of the IRE1α-XBP1 branch on the survival of CTCs *in vivo*.

## Role of the UPR on Colonization and Dormancy

CTCs surviving in the circulation arrive at the bone marrow vasculatures and extravasate into bone marrow parenchyma. It is still unclear whether this process is completed by passive entry due to the discontinuous endothelium of bone marrow sinusoids or if any other pathway actively involved (6, 7, 93). Compared with other organs, the bone is unique for its mineral content, enriched vasculatures, low oxygen level, high local Ca^2+^ concentration, and acidosis (94). As a result, the newly arrived tumor cells are challenged in many aspects (5, 6). Meanwhile, DTCs in bone remain dormant state in a variable period, which is critical for their survival, adaptation, escaping systemic treatments, and final outgrowth (6, 9, 94).

The hostile microenvironment (e.g., hypoxia) in the bone may disrupt ER protein folding; therefore, UPR pathways are expected to be upregulated in these DTCs. Indeed, UPR target genes are upregulated in dormant cancer cells from patients and mouse models (95–99). In the bone marrow of breast cancer patients, both GRP78/BiP and GRP94 are selectively highly expressed by bone marrow (BM) DTCs (98). Interestingly, UPR target genes are also overexpressed in cells derived from bone marrow DTCs compared with those from primary tumors (98, 100). These studies suggest that UPR upregulation is a stable trait for BM DTCs.

This trait may arise from the selection of pre-existing UPR positive subpopulation by the hostile microenvironment (and treatment, see discussion below) from the heterogenous cancer cell population, adaptation of the survived cancer cells to the microenvironment, or both. Nevertheless, these UPR genes are thought to confer a survival advantage to DTCs within the bone microenvironment because cell lines derived from BM DTCs are more resistant to glucose and oxygen deprivation *in vitro*. Studies in the head and neck cancer cell line HEp3 indicated that p38 plays a critical role in the induction and maintenance of tumor dormancy (95–97, 101). Interestingly, p38 activates all three branches of UPR in the dormant HEp3 cells, which contributes to the survival of cancer cells under glucose deprivation or chemotherapeutic treatments. Meanwhile, the PERK pathway inhibits the translation of cyclin D1/D3 and CDK4 in these cells, thereby arresting the cells in the G0-G1 phase. These studies support a causal role for the UPR in the establishment of dormancy (95–97). The upregulation of UPR genes are also found in dormant pancreatic ductal adenocarcinoma DTCs from lives of patient samples and mouse model (99). Collectively, these data indicate that UPR activation may be a common strategy utilized by cancer cells to enter dormancy and promote their survival. Further studies would be worthwhile to follow up on these impressive results and answer the following questions: (1) what triggers and/or maintains UPR signaling in dormant cancer cells in which overall protein synthesis is attenuated (101); (2) can UPR activation contribute to the dormant state of bone marrow DTCs *in vivo*, and if so, how; (3) what determines the pro-survival or pro-apoptotic effects of UPR activation in these cells; and (4) can the inhibition of the UPR promote DTCs death or sensitize them to therapies targeting proliferating cells.

## Role of the UPR on the Reactivation and Outgrowth of DTCs

Our current knowledge about the reactivation process of dormant DTCs, particularly in bone, is limited (4–6, 102). The autonomous traits of tumor cells alone cannot explain the asynchronized relapse of metastases after a long latency. Alternatively, local stimulation of the microenvironments may awaken dormant tumor cells. In bone, osteoclasts are key players in the microenvironmental support of osteolytic breast cancer cell growth and bone destruction. The upregulation of vascular cell adhesion molecule 1 (VCAM-1) in tumor cells promotes the transition from indolent micrometastasis to overt metastasis in breast cancer (103). DTCs with high VCAM-1 recruit integrin α4β^+^ osteoclast progenitors and induce local osteoclast activity. Therapeutically targeting the VCAM-1–integrin a4 interaction effectively inhibits the progression of bone metastasis and preserves bone structure in mouse models (103). Osteoblasts are another cell type found in the remodeling bone environment. It has been suggested that cancer cells interact with osteogenic cells through E-cadherin/N-cadherin and gap junctions and such interaction promotes early-stage bone colonization and outgrowth (104, 105). In multiple myeloma, XBP1 is required for the expression of VCAM-1, IL6, and RANKL and promotes osteolytic outgrowth (106). Given that XBP1 is one of the top transcription factors enriched in bone metastases compared with primary tumors and metastases in other organs (105), additional research is necessary to determine whether XBP1 regulates VCAM-1 in bone metastasis and promotes outgrowth.

Similarly to metastases in other organs, the immune system is absolutely critical in regulating the outgrowth of bone metastasis (94). In clinical practice, donor-derived cancer develops on rare occasions in immune-suppressed recipients who have received organs from cancer survivors (disease free for more than 10 years) or donors without diagnosable cancer at the time of transplantation (107–109). These observations suggest that the competent immune system may hold disseminated tumor cells in an asymptomatic state. Indeed, a higher ratio of CD56^+^ CD8^+^ T cells and memory CD4^+^ T cells were found in DTC-present bone marrow samples than in DTC-free samples in breast cancer patients (110). In a mouse model of spontaneous bone metastasis, the restoration of interferon regulatory factor 7 (Irf7) suppresses bone metastases through interferon signaling, whereas the deficiency of T and NK cell responses accelerates breast cancer bone metastases (111). A possible interpretation of these results is that cancer cell proliferation is balanced by immune-mediated cancer cell death (4, 112). The bone marrow is occupied by diverse immune cells including neutrophils (113–115). With age, hematopoietic stem cells gradually lose their self-renewal and regeneration capacity and are biased to differentiate into myeloid lineage including monocytes (giving rise to macrophages and dendritic cells), granulocytes (giving rise to basophils, neutrophils, and eosinophils), and megakaryocytes (116–118). This leads to an aged-related decline of the immune response (referred to as immunosenescence) and chronic, sterile, low-grade inflammation (named “inflamm-aging”) in older adults (119, 120). Inflammation is linked to the relapse of breast cancer (121). Sustained experimental inflammation and the accompanying formation of neutrophil extracellular traps in the lungs was found to convert dormant breast cancer cells to aggressive lung metastases in mice. Mechanistically, the neutrophil extracellular traps associated protease neutrophil elastase and matrix metalloproteinase 9 sequentially cleaves the ECM component laminin, leading to laminin remodeling. The remodeled laminin activates α3β1-FAK signaling in dormant cancer cells to induce their reactivation (122). As discussed above, XBP1 promotes neutrophils into immunosuppressive cells. In addition, the inhibition of the IRE1α RNase activity downregulates the expression and secretion of CXCL1 in multiple breast cancer cell lines (23), indicating the possibility that IRE1α promotes neutrophil recruitment by activating CXCL1. Furthermore, the IRE1a-XBP1 pathway is required for neutrophil extracellular trap formation during infection (123) Overall, the IRE1a-XBP1 pathway is known to promote neutrophil recruitment and function. Nevertheless, additional investigation is necessary to test whether neutrophils contribute to DTC reactivation in bone and whether/how the IRE1α-XBP1 pathway is involved in this process.

Dendritic cells (DCs) are responsible for the presentation of tumor antigens to T cells and initiation of the antitumor response (124). Activated T cells, especially cytotoxic CD8+ T cells and CD4+ T helper 1 cells, attack and destroy the target tumor cells (125). However, these processes are often inhibited by tumor cells via multiple strategies including at least by silencing the antigen presentation (hiding major histocompatibility complex I (MHCI) or making dendritic cells (DCs) dysfunctional), T-cell dysfunction, and the establishment of an immunosuppressive tumor microenvironment by myeloid-derived suppressor cells (MDSCs) (124–126). In contrast to the essential role of the IRE1α-XBP1 pathway in the physiology of antigen presentation cells under homeostatic conditions (127, 128), a study by the Laurie Glimcher's laboratory uncovered XBP1s as a critical driver of tumor-associated dendritic cell (tDC) dysfunction in the ovarian cancer microenvironment (129). IRE1α activation of XBP1s, stimulated by lipid peroxidation byproducts in tDCs, leads to abnormal lipid accumulation and subsequent inhibition of the antigen-presenting capacity of tDCs. Accordingly, DC-specific XBP1 inhibition restores their immunostimulatory capacity and extends survival in tumor-bearing mice. In addition, targeting the IRE1α-XBP1 pathway benefits T-cell function directly in the ovarian cancer microenvironment by increasing mitochondrial respiration activity (130) and attenuating cholesterol-induced CD8^+^ T-cell exhaustion (131). The PERK downstream target *Chop* (encode by Ddit3) is highly expressed in tumor-associated MDSCs, and the depletion of Chop compromises the function of MDSCs and delays tumor growth (132). Therefore, inhibition of the IRE1α and PERK pathways could boost the immune response in multiple tumors.

Taken together, these recent findings suggest that ER stress is induced in tumor cells and infiltrated immune cells in the tumor microenvironment. Thus, it would be interesting to test whether the abovementioned functions of the UPR are specific to the tumor microenvironment studied or can be generalized to other cancer types and different metastatic organs including bone.

## Therapeutic Resistance and Metastatic-Related Morbidity

Metastatic cancer often represents a terminal illness and is the main cause of cancer death (133). Current treatments for metastatic lesions are essentially similar to those for the corresponding primary tumors, including chemotherapy, targeted therapy, hormone therapy, radiation therapy, and immunotherapy (4, 134). Unfortunately, therapeutic resistance often occurs (4) due to many mechanisms, including tumor dormancy, stem-like properties, EMT, and immune suppression as discussed above. In a mouse model of spontaneous lung metastases from mammary tumors, *IRE1*α expression was induced upon cyclophosphamide-mediated chemotherapy (135). This result is further supported by a study that reported that IRE1α RNase activity is induced upon paclitaxel treatment in TNBC cells (23). Importantly, the inhibition of IRE1α RNase activity increases paclitaxel-mediated tumor suppression and delays tumor relapse posttherapy (23). This is consistent with our recent finding that the inhibition of IRE1α RNase activity substantially enhances the efficacy of docetaxel-based chemotherapy in treating MYC-overexpressing primary tumors and lung metastases (26). In summary, hijacking and upregulation of the IRE1α-XBP1 pathway is one strategy tumor cells use to develop chemoresistance, yet further investigation is required on the detailed mechanisms about how this pathway is activated and how it leads to resistance.

Bone pain is one of the most frequent symptoms of bone metastases, impairing both life quality and expectancy (136). One of the extensively studied molecules that leads to bone pain is cyclooxygenase-2 (COX-2), which is the key enzyme in prostaglandin biosynthesis (136, 137). Prostaglandins bind to prostanoid receptors on sensory terminals, resulting in bone pain (136). Inhibition of COX-2 attenuates bone pain, tumor growth, and bone destruction in a mouse model (138). The two latter phenotypes can be explained by the fact that prostaglandins can also directly promote cancer cell proliferation and induce immunosuppression (137). Recently, the IRE1α-XBP1 pathway was identified as an important regulator in prostaglandin biosynthesis and pain management (139). In myeloid cells (including macrophages and monocytes), XBP1 directly activates the expression of *COX-2* and *mPGES-1*. Genetically or pharmacologically inhibition of the IRE1α-XBP1 pathway diminished pain-related behaviors in mouse models. Given the established functions of COX2/PGES-1 in pain and immunosuppression, this finding not only revealed a new therapeutic approach for attenuating pain behavior but also indicated an alternative explanation how the IRE1α-XBP1 arm promotes immunosuppression.

## Conclusions and Future Directions

In the past decade, great strides have been made in bone metastasis research to enhance our understanding of this disease in both patients and experimental models. However, some key questions still remain unanswered. What triggers DTC dormancy and reawakening? How do DTCs evade immune cell surveillance? And ultimately, can we cure bone metastases? To address these questions, both conceptual and technological advances must be made. Improved models need to be developed that faithfully mimic the natural history of bone metastases in patients. The advancement in single-cell RNA sequencing has broadened our knowledge about the heterogeneity of cancer and bone marrow niche cells (114, 115, 140). This technique alone or together with the metastatic-niche labeling strategy (141) will shed new light on the biology of bone metastases and may identify new therapeutic targets.

The activation of the UPR has been demonstrated to endow cancer cells with tumorigenic, metastatic, and drug-resistant capacities and provide tumors with an immunosuppressive microenvironment. Given the convincing underlying mechanisms discovered and the exciting therapeutic results so far, it would be very promising to translate our current knowledge on the functions of the UPR in primary tumors to the study of bone metastases (Figure 3). Further studies are required to characterize the functions of the UPR in different steps of bone metastasis and in different cancer models. What are the driver events that induce/inhibit the UPR during bone metastasis? How does the UPR interplay with other signaling during this process? Can these stress responses in cancer cells be transmitted to niche cells to promote bone metastasis (142, 143)? Importantly, due to the immunosuppressive function of the UPR and the availability of multitarget drugs, it is conceivable to combine these inhibitors to various forms of cancer immunotherapy strategies to control bone metastases.

**Figure 3:** Potential connections between the UPR and bone metastasis. Schematic representation of the proposed effects of the UPR in bone metastasis by regulating indicated processes.

## Author Contributions

LX and XC: wrote the manuscript. WZ and XZ: contributed to the bone metastasis part. All authors contributed to the article and approved the submitted version.

## Conflict of Interest

The authors declare that the research was conducted in the absence of any commercial or financial relationships that could be construed as a potential conflict of interest.
